The article "Study on the Relationship between MMP-2, MMP-9 Gene Polymorphisms, and the Risk of Colorectal Cancer" was retracted in 2023. Reasons: unreliable results or conclusions; concerns about the data; concerns about the peer review; concerns about the citations.

# Study on the Relationship between MMP-2, MMP-9 Gene Polymorphisms, and the Risk of Colorectal Cancer

**DOI:** 10.1155/2022/7357160

**Published:** 2022-09-27

**Authors:** Su Peng, Maoliang Chen, Chunyun Wang, Changhua Liu, Kangning Luo, Lebin Yang

**Affiliations:** The Second Affiliated Hospital, Department of Gastrointestinal Surgery, Hengyang Medical School, University of South China, Hengyang, Hunan 421001, China

## Abstract

**Objective:**

The aim of the study is to explore the relationship between matrix metalloproteinase 2 (MMP-2) and matrix metalloproteinase 9 (MMP-9) gene polymorphisms and the risk of colorectal cancer.

**Methods:**

From January 2019 to December 2021, 308 patients with colorectal cancer in our hospital were selected to be included in the colorectal cancer group and 300 normal healthy people were included in the control group. We perform genotyping, compare the genotype frequencies between the colorectal cancer group and the control group, calculate the relationship between MMP-2 and MMP-9 gene polymorphisms and disease risk, and analyze the genotype distribution characteristics of colorectal cancer patients with different pathological stages and lymph node metastasis status. The expression levels of serum MMP-2 and MMP-9 in patients with different genotypes were compared.

**Results:**

The frequency of CC genotype and C gene at the MMP-2 gene−735 (C/T) locus in the colorectal cancer group was higher than that of the control group, and the frequency of TT genotype and T gene at MMP-9 gene−1562 (C/T) locus was a higher control group (*P* < 0.05). The comparison of genotype and gene frequency distribution of MMP-2 gene−1306 (C/T), −790 (T/G), and MMP-9 gene R668Q and P574R between the colorectal cancer group and the control group (*P* > 0.05); MMP-2 gene−735 (C/T) locus CC genotype and MMP-9 gene−1562 (C/T) locus TT genotype are dangerous genotypes for colorectal cancer. OR values were 1.490 (95% CI: 1.085–2.047), 1.519 (95% CI: 1.061–2.174); TNM stage III-IV, the proportion of CC genotype and TT genotype at MMP-9 gene−1562 (C/T) locus in patients with lymph node metastasis is higher than that without lymph node metastasis of TNM stage I-II patients (*P* < 0.05); MMP-2 gene in colorectal cancer patients. Serum MMP-2 levels in patients with CC genotype at 735 (C/T) locus were higher than those with CT + TT genotype, and serum MMP-9 levels in patients with TT genotype at MMP-9 gene−1562 (C/T) locus were higher CT + CC genotype patients (*P* < 0.05).

**Conclusion:**

The CC genotype at −735 (C/T) locus of the MMP-2 gene and the TT genotype at−1562 (C/T) locus of the MMP-9 gene are risk genotypes for the development of colorectal cancer.

The article "Study on the Relationship between MMP-2, MMP-9 Gene Polymorphisms, and the Risk of Colorectal Cancer" was retracted in 2023. Reasons: unreliable results or conclusions; concerns about the data; concerns about the peer review; concerns about the citations.

## 1. Introduction

Colorectal cancer, also known as colorectal cancer, is one of the most common digestive tract malignant tumors in my country. The statistical results of relevant data suggest [1] that the five-year survival rate of colorectal cancer can reach 90% if it is detected early and treated early. However, many countries still lack effective means of early screening, and less than 40% of patients are diagnosed early. The occurrence, invasion, and metastasis of colorectal cancer involve multiple pathophysiological processes, such as changes in the internal environment, gene mutations, abnormal cell pathways, and immune disorders [2].

(MMPs) are a group of important enzymes that can degrade ECM and BM, which can promote the invasion and metastasis of tumor cells and the formation of new blood vessels. Twenty-six kinds of MMPs have been found to degrade almost all extracellular matrix components, and they are the research hotspots of tumor invasion and metastasis mechanisms in recent years. Matrix metalloprotein-2 (MMP-2) and matrix metalloprotein-9 (MMP-9) are members of the matrix metalloproteinases (MMPs) family, which are the main enzymes that degrade the extracellular matrix. It can promote the infiltration of tumor cells to surrounding tissues along the basement membrane and accelerate the formation and spread of tumors [3]. Due to biological diversity, human similarities and differences, and multistage carcinogenicity, different individuals have different susceptibility to carcinogen exposure, and genetic polymorphism is an important reason for individual differences in response to environmental factors [4]. There are polymorphisms in human MMP-2 and MMP-9 genes, and their genetic variation affects the expression, structure, and function of MMP-2 and MMP-9, as well as their biological activities. Studies have found that MMP-9 is one of the proteins most closely related to colorectal malignancies in the MMP family. Its main function is to degrade collagen IV and V, gelatin, and elastic fibers in the extracellular matrix (ECM), and induce cancer cells. In the process of ECM degradation, MMP-9 releases a large amount of stored vascular endothelial growth factor (VEGF), thus inducing the formation of new blood vessels, providing nutrients for tumor cells and accelerating blood transmission. Therefore, detecting the expression of MMP-9 in tumor tissue is helpful for judging the degree of progression of colorectal cancer and has guiding significance for evaluating the prognosis. This study analyzed the relationship between MMP-2 and MMP-9 gene polymorphisms and colorectal cancer susceptibility, aiming to detect susceptible people early and take corresponding measures to reduce the risk of the disease. The report is as follows.

The article "Study on the Relationship between MMP-2, MMP-9 Gene Polymorphisms, and the Risk of Colorectal Cancer" was retracted in 2023. Reasons: unreliable results or conclusions; concerns about the data; concerns about the peer review; concerns about the citations.

## 2. Objective and Methods

### 2.1. General Information

A total of 308 colorectal cancer patients in our hospital from January 2019 to December 2021 were selected and included in the colorectal cancer group. Among them, 160 were males and 148 were females; 137 cases were <60 years old and 171 cases were ≥60 years old; tumor site: 142 cases of colon, 166 cases of the rectum; degree of differentiation: 177 cases of moderate and well differentiated, 131 cases of poor differentiation; TNM Stage: 169 cases of stage I-II, 139 cases of stage III-IV, lymph node metastasis: no 186 cases, 122 cases.

The inclusion criteria were as follows: (1) primary colorectal cancer, diagnosed by pathology; (2) age ≥ 18 years old; (3) have not received radiotherapy, chemotherapy, and biological therapy before enrollment; and (4) approved by the hospital ethics committee and the patients and their families agreed to sign.

The exclusion criteria were as follows: (1) combined with other serious tumor diseases; (2) combined with autoimmune diseases; (3) combined mental illness; (4) complicated with a history of severe organic heart, liver, and lung disease; (5) received antitumor therapy such as radiotherapy and chemotherapy before enrollment; (6) pregnant and lactating women; and (7) unwilling patients. Another 300 healthy subjects were selected and included in the control group.

### 2.2. Methods

#### 2.2.1. Collection of General Data

The basic clinical data of the research subjects were collected through profile questionnaires, a literature review, combined with clinical practice, and pretest corrections were performed. The survey contents included demographic characteristics, personal disease history, family history, exposure history of major risk factors in the past year (including dietary habits, physical exercise, and lifestyle), smoking (≥5 cigarettes per day and more than 1 year), alcohol consumption (>2 times/week, beer consumption >500 mL/time or rice wine consumption >250 mL/time or liquor consumption >50 mL/time), frequent consumption of spicy food (average > 3 times)/week), frequent consumption of pickled barbecued food (average > 2 times)/week), regular physical exercise (average > 4 times/week). Professionally trained and qualified investigators conduct face-to-face investigations, check in real time, and logically check the input data. If there are omissions or errors, they will be filled and corrected.

#### 2.2.2. MMP-2 and MMP-9 Gene Polymorphism Detection

The polymerase chain reaction-restriction fragment length polymorphism (PCR-RFLP) technique was used to detect and detect MMP-2 (−1306 (C/T) locus, −735 (C/T) locus, −790 (T) locus/G) locus) and MMP-9 (−1562 (C/T) locus, R668Q locus, P574R locus) gene polymorphisms. (1) Specimen collection: 5 mL of fasting venous blood was drawn from the included subjects, mixed with EDTA evenly, and stored at −80°C. (2) Genomic DNA extraction: The genome was extracted using a blood genome kit (Beckman AMPurea XPDNA), DNA was extracted from leukocytes, dissolved in double distilled water, and after the purity of the samples was qualified, the samples were stored at −80°C for testing. (3) Primer design and synthesis: primer design (Sequenom, USA), primer synthesis (Chengdu Synthetic Biotechnology Co., Ltd.). Primer sequence: MMP-2: ① 1306 (C/T) locus: upstream: 5′-CTTCCTAGGCTGGTCCTTAC-3′, downstream: 5′-AGACCTGAAGAGCTAAAGACG-3′; ② -735 (C/T): Upstream: 5′-ATAGGGTAAACCTCCCCACATT-3′, Downstream: 5′-GGTAAAATGAGGCTGAG ACCTG-3′; ③ 790 (T/G): upstream: 5′-CACTGGTGGGTGCTTCCTTTAAC-3′, downstream: 5′-TGAGATAGAAATTGGGCAAGACTGGTTTACTA-3′. MMP-9: ① 1562 (C/T): Upstream: 5′-GCCTGGCACATAGTAGGCCC-3′, Downstream: 5′-TTCCTAGCCAGCCGGCATC-3′; ② R668Q: Upstream: 5′-ACACGCACGACGTC TTCC AGTATC-3′, downstream: 5′-GGGGCATTTGT TTCCATTTCCA-3′; ③ P574R: Upstream: 5′-GCTGGACTCGGTCTTTGAGGATC-3′, Downstream: 5′-TTGAGCCTCCTTGA CTGATGGG-3′. (4) Genotyping analysis: ① Amplification: PCR amplification reaction volume is 25 *μ*L, including template (6 *μ*L), upstream and downstream primers (1 *μ*L each), 12.5 *μ*L 2 × Taq PCR Master Mix, 4.5 *μ*L deionized water, PCR amplification reaction parameter settings: pre-denaturation (95°C, 5 min), denaturation (95°C, 30s), annealing (62°C, 30s), extension (72°C, 1 min), 35 cycles, and final extension 72°C, 5 min. ② Genotyping and sequencing: The enzyme digestion reaction system is 20 *μ*L, including PCR amplification products 12 *μ*L, Hinf I endonuclease 2.0 *μ*L, 10× restriction endonuclease buffer 2.0 *μ*L, deionized water 4.0 *μ*L. After 30 min in a water bath at 37°C, the digested products were electrophoresed on a 2.5% agarose gel, and their genotypes were analyzed by a gel imaging analysis system.

The article "Study on the Relationship between MMP-2, MMP-9 Gene Polymorphisms, and the Risk of Colorectal Cancer" was retracted in 2023. Reasons: unreliable results or conclusions; concerns about the data; concerns about the peer review; concerns about the citations.

#### 2.2.3. Detection of Serum MMP-2 and MMP-9 Levels

4 ml of fasting venous blood was centrifuged at 3000 r/min for 10 min and the supernatant was taken. MMP-2 and MMP-9 were detected by an enzyme-linked immunosorbent assay. The microplate reader was operated according to the kit instructions.

### 2.3. Statistical Methods

SPSS 22.0 statistical software was used for data statistics; count data were expressed as percentages (%) and comparisons between groups were performed using the *χ*^2^ test or Fisher's exact test. Measurement data are expressed as mean ± standard deviation. Independent sample *t* test comparison between groups. The logistic regression was used to analyze the risk factors for colorectal cancer. *P* < 0.05 means the difference is statistically significant.

## 3. Results

### 3.1. Comparison of General Data between the Colorectal Cancer Group and Control Group

There was no statistical difference between the colorectal cancer group and the control group in terms of gender, age, BMI index, smoking, irregular diet, and physical exercise (*P* > 0.05). The colorectal cancer group had a higher proportion of family history, drinking alcohol, and frequent consumption of pickled food than the control group (*P* < 0.05) as shown in Table 1.

### 3.2. Comparison of MMP-2, MMP-9 Genotype, and Frequency Distribution between the Colorectal Cancer Group and Control Group

Colorectal cancer group and control group MMP-2 and MMP-9 genes−1306 (C/T), −735 (C/T), −790 (T/G), and −1562 (C/T), R668Q, P574R. The genotype distribution of points was in accordance with the Hardy–Weinberg equilibrium (*P* > 0.05).

The CC genotype and C gene frequency of the MMP-2 gene −735 (C/T) locus in the colorectal cancer group were higher than those of the control group, and the TT genotype and T gene frequency of the MMP-9 gene −1562 (C/T) locus were higher than those of the control group. Control group (*P* < 0.05); Comparison of genotype and gene frequency distribution of MMP-2 gene −1306 (C/T), −790 (T/G) and MMP-9 gene R668Q, P574R in colorectal cancer group and control group (*P* > 0.05) as shown in Table 2.

### 3.3. Analysis of Risk Factors Affecting the Occurrence of Colorectal Cancer

Using a generalized model, logistic regression analysis was performed on the above items with statistically significant differences and assigned values, family history of colorectal cancer (no = 0, yes = 1), alcohol consumption (no = 0, yes = 1), frequent consumption of pickled food and grilled food (no = 0, yes = 1), MMP-2-735 (C/T) genotype (CT or TT type = 0, CC type = 1), MMP-9-1562 (C/T) genotype (CC or CT type = 0, TT type = 1). Logistic regression analysis showed that family history of colorectal cancer, alcohol consumption, frequent consumption of pickled barbecued food, MMP-2 gene −735 (C/T) locus CC genotype, and MMP-9 gene −1562 (C/T) locus TT genotype are an independent risk factors for colorectal cancer. MMP-2 gene −735 (C/T) locus CC genotype and MMP-9 gene −1562 (C/T) locus TT genotype are risk genotypes for colorectal cancer. The OR values were 1.490 (95% CI: 1.085–2.047) and 1.519 (95% CI: 1.061–2.174), respectively as shown in Table 3.

### 3.4. Comparison of MMP-2 and MMP-9 Genotype and Frequency Distribution in Colorectal Cancer Patients with Different Pathological Features

In TNM stage III-IV, the proportion of CC genotype at−735 (C/T) locus of MMP-2 gene and TT genotype at −1562 (C/T) locus of MMP-9 gene in patients with lymph node metastasis was higher than that in TNM stage I-stage II patients without lymph node metastasis (*P* < 0.05) as shown in Table 4.

The article "Study on the Relationship between MMP-2, MMP-9 Gene Polymorphisms, and the Risk of Colorectal Cancer" was retracted in 2023. Reasons: unreliable results or conclusions; concerns about the data; concerns about the peer review; concerns about the citations.

### 3.5. Comparison of Serum MMP-2 and MMP-9 Levels in Colorectal Cancer Patients with Different MMP-2 and MMP-9 Genotypes

Among 308 patients with colorectal cancer, the serum MMP-2 level in patients with CC genotype at MMP-2 gene−735 (C/T) locus was (139.05 ± 32.06) ng/mL higher than that in patients with CT + TT genotype (119.75 ± 27.44) ng/mL (*P* < 0.05). MMP-9 gene−1562 (C/T) locus patients with TT genotype serum MMP-9 level (179.18 ± 39.51) ng/mL higher than CT + CC genotype patients (151.62 ± 31.24) ng/mL (*P* < 0.05) as shown in Table 5.

## 4. Discussion

In the early stages of colorectal cancer, there may be no obvious clinical symptoms. With the passage of time and the continuous growth of the tumor, changes in bowel habits and symptoms of abdominal pain may occur, and further aggravation may cause systemic changes in patients [5]. With the rapid development of cellular and molecular biology research at this stage, the occurrence, development, invasion, metastasis mechanism, and treatment of malignant tumors have become a hotspot in clinical research.

MMPs are a group of zinc ion-dependent endopeptidases, which can degrade almost all extracellular matrix and vascular basement membrane, participate in embryonic development and tissue modeling, and are also proteolytic enzymes involved in tumor cell invasion and metastasis [6]. Under pathological conditions, MMPs not only break through the matrix barrier by degrading the matrix membrane and surrounding tumor matrix to promote tumor invasion and metastasis but also stimulate tumor growth and spread by promoting endothelial cell migration and angiogenesis [7]. Both MMP-2 and MMP-9 are closely related factors in the MMP family. Among them, the MMP-2 gene is located on human chromosome 16q21, secreted in the form of zymogen, and activated after hydrolysis, which can degrade the components of the intercellular matrix, and can also destroy the integrity of the basement membrane, allowing cancer cells to infiltrate the damaged extracellular space around the substrate. MMP-9 is located on chromosome 20q11.2-q13.1, can degrade extracellular matrix gelatin, various collagens, elastic fibers, etc., and plays an important role in tumor invasion and metastasis [8,9].

Sequence analysis of the MMP-2 gene showed that [10], the promoter region of the MMP-2 gene contains a variety of cis-acting elements such as AP-1, SP-1 and AP-2, suggesting that there are multiple transcription factors in the transcription process of the MMP-2 gene participation. In this study, −1306 (C/T) and −735 (C/T) are located upstream of the MMP-2 transcriptional start point, which may alter protein expression by changing gene transcriptional activity. Studies have shown that the risk of lung cancer in Chinese people with −1306CC genotype is 1.6 times higher than that of the CT or TT genotypes, and the risk of oral squamous cell carcinoma is 2 times higher [11]. However, in this study, there was no significant difference in the genotype distribution of the −1306 (C/T) locus between the colorectal cancer group and the control group. The −1306 (C/T) locus gene polymorphism did not affect the risk of colorectal cancer. The impact mechanism of colorectal cancer is complex, and many genes are involved in the occurrence of the disease. A single gene has little effect, and different stimuli may have different effects [12]. In this study, the frequency of the CC genotype and C allele at the −735(C/T) locus in the colorectal cancer group was higher than those in the control group. Logistic regression analysis showed that the CC genotype was an independent risk factor for colorectal cancer susceptibility, and the CC gene The risk of colorectal cancer in patients with this genotype was 1.490 times that of the CT + TT genotype. To analyze the possible reasons, the T ⟶ C change at the −735 (C/T) locus in the MMP-2 promoter region destroyed the binding locus of the transcription factor Sp1, significantly reduced the promoter activity, and affected the expression level of MMP-2. This study also showed that the expression level of serum MMP-2 in individuals with CC genotype was higher than that in individuals with TT or CT genotype, further indicating that CC genotype at −735 (C/T) locus can alter gene transcriptional activity and affect MMP-2 expression, which in turn affects tumorigenesis. Some researchers found that patients with TT or CT genotype at the MMP-2 gene−735 locus in small cell lung cancer had longer survival and a lower risk of death than those with CC genotype [13]. In this study, the relationship between the −735(C/T) locus genotype and the clinicopathological characteristics of colorectal cancer was compared and analyzed. The results showed that the −735(C/T) locus had a higher proportion of patients with high clinical stage and lymph node metastasis with CC genotype. Indicating that the −735(C/T) locus CC genotype increases the risk of colorectal cancer disease development and metastasis. At the same time, this study showed that MMP-2 gene−790 (T/G) was not associated with the risk of colorectal cancer.

The article "Study on the Relationship between MMP-2, MMP-9 Gene Polymorphisms, and the Risk of Colorectal Cancer" was retracted in 2023. Reasons: unreliable results or conclusions; concerns about the data; concerns about the peer review; concerns about the citations.

In addition, this study selected MMP-9 gene −1562 (C/T), Q279R, P574R, a total of 3 SNP loci, to study in the colorectal cancer group and the control group. Nascimento et al. [14] pointed out that MMP-9−1562 (C/T) gene polymorphism is associated with aortic aneurysm, colorectal cancer, lung cancer and so on. This study also showed that the TT genotype frequency and T allele frequency of the MMP-9 gene −1562 (C/T) locus in the colorectal cancer group were higher than those in the control group, which was consistent with the above research results. With genotype CC and CT as reference, the adjusted OR (95% CI) of genotype TT was 1.519 (95% CI: 1.061–2.174), which can be considered as an MMP-9 gene −1562 (C/T) locus polymorphism, which is related to the occurrence of colorectal cancer, and TT genotype may increase the risk of colorectal cancer susceptibility. Among colorectal cancer patients, the frequency of the TT genotype was higher in patients with stage III-IV than in patients with stage I-II, and it was found that TT genotype carriers were more prone to lymph node metastasis than CC + CT genotypes. The study of Walter et al. [15] showed that tumor formation, metastasis, and invasion were inhibited in MMP-9-deficient transgenic mice. After transplantation of MMP-9-expressing bone marrow cells, tumor formation and invasiveness were restored. This shows that MMP-9 contributes to tumor cell invasion and metastasis. In this study, the differences in serum MMP-9 expression levels in colorectal cancer patients with different genotypes at the −1562 (C/T) locus were compared. The results showed that the expression level of serum MMP-9 in patients with TT genotype was higher than that of CT + CC genotype, and the change of C ⟶ T at −1562 (C/T) locus could promote the expression of MMP-9 and mediate the occurrence and development of colorectal cancer. In this study, a case-control study method was used to analyze the relationship between the MMP-9 gene P574R polymorphism and R668Q polymorphism and the risk of colorectal cancer. The results showed that P574R and R668Q gene polymorphisms were not associated with the risk of colorectal cancer.

The disadvantages of this study are that race was not excluded as a confounder, the results of this study may not be generalizable to patients outside the region, and clinical data such as patient survival and sensitivity to chemoradiotherapy were not analyzed. The follow-up sample will be expanded to allow for further follow-up studies.

In conclusion, MMP-2 gene −735 (C/T) locus CC genotype and MMP-9 gene −1562 (C/T) locus TT genotype are risk genotypes for the occurrence and development of colorectal cancer. The detection of related gene polymorphisms can detect the susceptible population of colorectal cancer early and take corresponding intervention measures as soon as possible to reduce the risk of the disease.

The article "Study on the Relationship between MMP-2, MMP-9 Gene Polymorphisms, and the Risk of Colorectal Cancer" was retracted in 2023. Reasons: unreliable results or conclusions; concerns about the data; concerns about the peer review; concerns about the citations.

## Figures and Tables

**Table 1:** Comparison of general information between the colorectal cancer group and control group.

Indexes		Number of cases (*n*)	Colorectal cancer group (*n* = 308)	Control group (*n* = 300)	*χ* ^2^	*P*
*Gender*	Male	310	160	150	0.231	0.631
	Female	298	148	150		
*Age (year)*	<60	267	137	130	0.081	0.776
	≥60	341	171	170		
*BMI index (kg/m* ^*2*^ * )*	<18.5	55	30	25	0.587	0.746
	18.5–23.9	485	242	243		
	>23.9	68	36	32		
*Family history of colorectal cancer*	Yes	32	26	6	12.647	<0.001
	No	576	282	294		
*Smoking*	Yes	193	101	92	0.317	0.574
	No	415	207	208		
*Drinking alcohol*	Yes	107	65	42	5.289	0.022
	No	501	243	258		
*Irregular diet*	Yes	134	73	61	1.003	0.317
	No	474	235	239		
*Regular consumption of marinated/barbecued food*	Yes	114	69	45	5.467	0.019
	No	494	239	255		
*Regular consumption of spicy food*	Yes	105	59	46	1.554	0.213
	No	503	249	254		
*Regular physical activity*	Yes	287	139	148	1.077	0.299
	No	321	169	152		

**Table 2:** Comparison of MMP-2 and MMP-9 genotype and frequency distribution between the colorectal cancer group and control group.

Indexes	Genetic locus			*Colorectal cancer group (n* *=* *308)*		*Control group (n* *=* *300)*		*χ* ^2^	*P*
				Number of cases	Frequency (%)	Number of cases	Frequency (%)		
MMP-2	Genotype	−1306 (C/T)	CC	243	78.90	226	75.33	1.385	0.500
			CT	62	20.13	69	23.00		
			TT	3	0.97	5	1.67		
		−735 (C/T)	CC	206	66.88	167	55.67	9.026	0.011
			CT	86	27.92	118	39.33		
			TT	16	5.19	15	5.00		
		−790 (T/G)	TT	235	76.30	226	75.33	0.182	0.913
			TG	69	22.40	69	23.00		
			GG	4	1.30	5	1.67		
	Gene frequencies	−1306 (C/T)	C	548	88.96	521	86.83	1.295	0.255
			T	68	11.04	79	13.17		
		−735 (C/T)	C	498	80.84	452	75.33	5.401	0.020
			T	118	19.16	148	24.67		
		−790 (T/G)	T	539	87.50	521	86.83	0.121	0.728
			G	77	12.50	79	13.17		

MMP-9	Genotype	−1562 (C/T)	CC	169	54.87	205	68.33	13.764	0.001
			CT	124	40.26	90	30.00		
			TT	15	4.87	5	1.67		
		R668Q	RR	291	94.48	276	92.00	1.528	0.466
			RQ	13	4.22	19	6.33		
			QQ	4	1.30	5	1.67		
		P574R	PP	275	89.29	277	92.33	1.809	0.405
			PR	26	8.44	19	6.33		
			RR	7	2.27	4	1.33		
	Gene frequencies	−1562 (C/T)	C	452	73.38	500	83.33	13.871	<0.001
			T	154	25.00	100	16.67		
		R668Q	R	595	96.59	571	95.17	1.564	0.211
			Q	21	3.41	29	4.83		
		P574R	P	576	93.51	573	95.50	2.320	0.128
			R	40	6.49	27	4.50		

**Table 3:** Analysis of risk factors affecting the occurrence of colorectal cancer.

Factor	Regression coefficients (*β*)	Standard error	Wald *χ*^2^ value	*P* value	OR value	95% CI
Family history of colorectal cancer	1.022	0.391	6.832	0.009	2.779	1.291–5.980
Drinking alcohol	0.506	0.198	6.531	0.011	1.659	1.125–2.445
Regular consumption of marinated/barbecued food	0.794	0.250	10.087	0.002	2.212	1.355–3.611
MMP-2-735 (C/T) gene type	0.399	0.162	6.066	0.014	1.490	1.085–2.047
MMP-9-1562 (C/T) gene type	0.418	0.183	5.217	0.023	1.519	1.061–2.174

The article "Study on the Relationship between MMP-2, MMP-9 Gene Polymorphisms, and the Risk of Colorectal Cancer" was retracted in 2023. Reasons: unreliable results or conclusions; concerns about the data; concerns about the peer review; concerns about the citations.

**Table 4:** Comparison of MMP-2 and MMP-9 genotype and frequency distribution in patients with colorectal cancer with different pathological characteristics.

Clinicopathological features		Number of cases	*MMP-2*		*χ* ^2^	*P*	*MMP-9*		*χ* ^2^	*P*
			(−735(C/T))				(−1562(C/T))			
			CC	CT + TT			TT	CT + CC		
			(*n* = 206)	(*n* = 102)			(*n* = 15)	(*n* = 293)		
TNM	Phase I-II	169	103	66	5.958	0.015	4	165	5.065	0.024
Staging	Phase III-IV	139	103	36			11	128		
Lymph node metastasis	No	186	116	70	4.327	0.038	5	181	4.825	0.028
	Yes	122	90	32			10	112		

**Table 5:** Comparison of serum MMP-2 and MMP-9 levels in colorectal cancer patients with different MMP-2 and MMP-9 genotypes.

Detection indicator	*MMP-2*		*T*	*P*	*MMP-9*		*T*	*P*
	(−735 (C/T))				(−1562 (C/T))			
	CC	CT + TT			TT	CT + CC		
	(*n* = 206)	(*n* = 102)			(*n* = 15)	(*n* = 293)		
MMP-2	139.05 ± 32.06	119.75 ± 27.44	5.207	<0.001	—	—	—	—
MMP-9	—	—	—	—	179.18 ± 39.51	151.62 ± 31.24	3.287	0.001

## Data Availability

The data used and/or analyzed during the current study are available from the corresponding author.
